The article "Detection and Diagnostic Value of Cytokines in Serum of Children with Acute Viral Encephalitis" was retracted in 2023. Reasons: signs of a paper mill; suspected computer-generated content; unreliable results or conclusions; lack of ethics approval or compliance.

# Detection and Diagnostic Value of Cytokines in Serum of Children with Acute Viral Encephalitis

**DOI:** 10.1155/2022/9997531

**Published:** 2022-09-27

**Authors:** Na Zhang, Jing Li, Xiaojing Yan, Weixiao Liu

**Affiliations:** The Third Department of Pediatrics, Xingtai People's Hospital, Xingtai 054000, China

## Abstract

Acute viral encephalitis is one of the serious infectious diseases. In order to analyze the diagnostic efficacy of serum procalcitonin (PCT), C-reactive protein (CRP), and S100B protein in acute viral encephalitis, a total of 100 children with acute viral encephalitis from July 2019 to December 2021 are selected and included in the viral encephalitis group. The results show that S100B protein model has high specificity and sensitivity and is simple to operate. It provides new ideas and directions for differential diagnosis, improvement, and optimization of relevant clinical diagnosis and treatment schemes and has high clinical value.

## 1. Introduction

Acute viral encephalitis is a serious infectious disease, which is related to children's central nervous system disease. Usually, cerebrospinal fluid extraction is performed to expand the relevant pathological examination. However, this study found that the detection method has certain limitations. For a long time, the positive rate of pathogen culture detected by cerebrospinal fluid analysis is low. To some extent, it affects its efficacy in clinical differentiation and diagnosis of acute viral encephalitis [1, 2]. It should be noted that acute viral encephalitis occurs and develops rapidly, during which the children's central nerve cells are affected by a variety of viruses, resulting in the damage of normal cells and the secretion of a large number of inflammatory factors [3, 4]. In order to further improve the clinical differential diagnosis efficiency of acute viral encephalitis, the purpose of this study is to analyze the expression of serum cytokines in children with acute viral encephalitis, explore its diagnostic value, and analyze the relationship between the development of cases and the degree, so as to provide some data support for the diagnosis of children with viral encephalitis.

The rest of this paper is organized as follows.  Section 2 discusses relevant research and summary analysis, followed by the patient's information and research methods in Section 3. The comparative analysis and data statistics are given in Section 4.  Section 5 concludes the paper with summary and future research directions.

## 2. Relevant Work

Clinical research data show that due to the influence of age and growth period, the central nervous system barrier system and related functions of children are not mature, and children have low immunity and high risk of being invaded by pathogenic bacteria because the incidence of central nervous system infection in children is also high [5, 6]. Viral encephalitis and bacterial meningitis are more common [7, 8]. In recent years, the epidemic trend of different viral encephalitis has appeared all over the world, indicating that with international communication, the virus has also begun to globalize, so it needs to be controlled [9]. Due to the differences in the pathogenesis factors, it is very important to carry out early diagnosis and select treatment plan, which plays a decisive role in its prognosis [10]. Its diagnosis mostly depends on positive bacterial culture or virus isolation, but its time consumption is too long, and the positive rate is relatively small, and there are also clinical cerebrospinal fluid atypical patients, so it brings great difficulties to its early diagnosis and has a serious impact on the clinical treatment effect of children. Due to early empiric antibiotic treatment, the positive rate of cerebrospinal fluid examination is low, especially the results of etiological examination, leading to missed diagnosis. Therefore, it is of great significance to explore sensitive biological markers for the accurate identification and diagnosis of acute viral encephalitis. PCT is a newly discovered inflammatory factor, which is often used in clinical diagnosis of infectious diseases. Under normal circumstances, the serum level of human PCT is low, and PCT is mainly produced by thyroid C cells [11–13]. This study shows that the PCT value of children with acute viral encephalitis is significantly higher than that of healthy children, and the index value shows a higher trend of expression with the aggravation of the severity of the children's disease. ROC curve is used to analyze the AUC of serum PCT level in the diagnosis of viral encephalitis in children (AUC = 0.781), which confirmed the high accuracy of serum PCT level. CRP is the main index reflecting the non-specific inflammatory response in the body, and it is usually increased when cardiac and cerebrovascular injury is serious, but only when the inflammatory response reaches a certain degree, CRP is detected to be positive [14–19]. This study shows that the CRP value of children with acute viral encephalitis is significantly higher than that of healthy children, and the index value would increase with the aggravation of the disease degree of children. ROC curve is used to analyze serum CRP level in diagnosing viral encephalitis in children. AUC = 0.755, indicating that serum CRP has a certain effect on differentiating children with acute viral encephalitis. S100B protein is an acidic calcium binding protein widely distributed in central and peripheral nerve tissues. The physiological level of S100B protein in the brain is mainly produced by astrocytes and acts on neurons and their surroundings. When S100B protein is overexpressed in glial cells, it can accelerate the deterioration of nervous system inflammation and lead to nervous system dysfunction. Clinical studies show that S100B protein is highly specific and sensitive to brain injury and can easily pass through the blood-brain barrier and sensitively reflect the degree of brain injury. At present, many studies show that the level of S100B protein increases significantly in the serum of patients with bacterial meningitis, and its diagnostic sensitivity and specificity are high, suggesting that S100B can be used as a marker of brain injury [20, 21].

## 3. Patient Information and Research Methods

### 3.1. Patients and Treatment

A total of 100 children with acute viral encephalitis admitted to our hospital from July 2019 to December 2021 are included in the viral encephalitis group, including 46 boys and 54 girls, aged from 1 to 12 years, with an average age of (6.02 ± 1.16) years, and 59 mild children and 41 severe children, with the course of disease ranging from 1 to 7 days. In addition, a total of 58 children suspected of intracranial infection who received physical examination in our hospital during the same period and are confirmed as healthy and normal after clinical biochemical and cerebrospinal puncture and other routine examinations are included in the healthy control group, including 42 boys and 58 girls, aged from 1 to 13 years, with an average of (6.15 ± 1.03) years. There are no significant statistical differences in baseline data such as gender and age between the two groups (all *P* > 0.05), which confirmed that the comparison between groups is scientific and reasonable.

Inclusion criteria for children were as follows: (1) the age range of children is 1–15 years; (2) all patients are diagnosed for the first time in our hospital; (3) the clinical symptoms and diagnostic results of the children all met the diagnostic criteria for viral encephalitis in the eighth edition of Zhufutang Practical Pediatrics; (4) complete clinicopathological data; and (5) the families of the children are informed of the study and signed the consent form.

Exclusion criteria for children were as follows: (1) poor clinical compliance and difficult to normally cooperate with the relevant investigation work of this study; (2) children complicated with suppurative meningitis, tuberculous meningitis, and other serious brain dysfunction diseases; and (3) children complicated with other acute infectious diseases.

### 3.2. Serum Factor Detection Method

5 mL of fasting peripheral venous blood is collected in both groups within 24 h after admission. Centrifuge is used for centrifugation, and the parameter is set at 3500 r/min with a centrifuge radius of 10 cm. The centrifuge operation lasted for 15 min. Serum PCT, CRP, and S100B proteins are detected by ELISA. The instrument is HED-SY96S microplate tester (purchased from Shandong Holder Electronic Technology Co. LTD.), and the kit is purchased from an American R&D company. The corresponding operations are performed strictly according to the kit instructions.

### 3.3. Observation Indicators

Firstly, the expression of serum PCT, CRP, and S100B proteins is compared. Secondly, the expression of serum PCT, CRP, and S100B proteins in children with acute viral encephalitis of different severity is compared. Thirdly, the diagnostic value of single and combined detection of serum PCT, CRP, and S100B protein indexes is analyzed. Finally, the correlation between the expression of serum PCT, CRP, and S100B protein and the severity of acute viral encephalitis is analyzed.

### 3.4. Statistical Processing

SPSS 26.0 software is used for statistical analysis of the data involved in this study, and the measurement data are verified. After confirming that the data are normally distributed, mean ± standard deviation $\left(\bar{x}\pm s\right)$ is used to represent the data differences between groups, and *t*-test is performed. The count data involved are represented by (*n*, %), and the differences between groups are analyzed by *x*^2^ test. Spearman correlation coefficient is used to analyze the correlation between the expression of PCT, CRP, and S100B protein and the severity of acute viral encephalitis. In this study, the diagnostic value of acute viral encephalitis is evaluated by ROC curve, and *P* < 0.05 proved that the difference is statistically significant.

## 4. Comparative Analysis and Data Statistics

### 4.1. The Expressions of Serum PCT, CRP, and S100B Proteins

The expression of serum PCT, CRP, and S100B protein in the viral encephalitis group increased significantly than that in the healthy control group (all *P* < 0.05), as shown in Table 1.

### 4.2. The Expression of Serum PCT, CRP, and S100B Proteins in Children with Acute Viral Encephalitis of Different Severity

A subgroup is established according to the severity of viral encephalitis. The children with mild encephalitis are included in the mild group (*n* = 59), and the children with severe encephalitis are included in the severe group (*n* = 41). The comparison of serum PCT, CRP, and S100B protein expressions between the two groups shows that with the aggravation of the severity of the disease, the values of serum indicators are significantly increased (all *P* < 0.05), as shown in Table 2.

### 4.3. Analysis of the Diagnostic Value of Single and Combined Detection of Serum PCT, CRP, and S100B Protein Indicators

ROC curve is used to analyze the diagnostic efficacy of serum PCT, CRP, and S100B protein indicators for acute viral encephalitis by single detection and combined detection, as shown in Table 3.

Figure 1 shows that the area under the curve of single detection is above 0.700, and the diagnostic efficacy of the combined detection of the three indicators is higher (AUC = 0.969).

### 4.4. Analysis of the Correlation between the Expression of Serum PCT, CRP, and S100B Protein and the Severity of Acute Viral Encephalitis

Spearman correlation coefficient analysis shows that the expression of serum PCT, CRP, and S100B protein is significantly positively correlated with the severity of acute viral encephalitis (all *P* < 0.05), as shown in Table 4.

## 5. Conclusions

The results of this study shows that the expression level of serum S100 protein in children with acute viral encephalitis is significantly increased compared with that in healthy children, and this index value would be higher with the aggravation of the severity of the disease in children. ROC curve is used to analyze serum CRP level in diagnosing viral encephalitis in children. AUC = 0.802. The area under the curve of the combined detection mode of the three serum factors is higher (0.969), suggesting that the combined detection of the three serum factors mentioned above has higher diagnostic efficacy for acute viral encephalitis in children. To sum up, serum PCT, CRP, and S100B detection method is a simple, rapid, more efficient clinical diagnosis and timely follow-up clinical method. It can determine acute viral encephalitis in serum by monitoring the above three indicators and can also use the above three indicators to evaluate and monitor the development of children's disease, which has high clinical significance.

## Figures and Tables

**Figure 1:** ROC diagram of PCT, CRP, and S100B protein and combined diagnosis of acute viral encephalitis.

**Table 1:** Comparison of serum PCT, CRP, and S100B protein expressions.

Group	PCT (ng/mL)	CRP (mg/L)	S100B protein (pg/mL)
Viral encephalitis group (*n* = 100)	0.78 ± 0.26	9.26 ± 2.78	0.36 ± 0.11
Healthy control group (*n* = 58)	0.42 ± 0.14	3.57 ± 0.84	0.22 ± 0.03
*T*	9.748	15.173	9.479
*P*	<0.001	<0.001	<0.001

**Table 2:** Comparison of serum PCT, CRP, and S100B protein expressions.

Group	PCT (ng/mL)	CRP (mg/L)	S100B protein (pg/mL)
Mild group (*n* = 59)	0.59 ± 0.16	7.48 ± 1.86	0.28 ± 0.05
Severe group (*n* = 41)	0.84 ± 0.29	11.32 ± 3.13	0.47 ± 0.16
*t*	−5.528	−7.681	−8.556
*P*	<0.001	<0.001	<0.001

**Table 3:** Value analysis of serum PCT, CRP, and S100B protein single index and combined diagnosis of acute viral encephalitis.

Indicators	AUC (95% CI)	Sensitivity (%)	Specificity (%)	About an index	Cutoff value
PCT (ng/mL)	0.781 (0.711 ∼ 0.850)	76.00	68.00	0.44	0.74
CRP (mg/L)	0.755 (0.678 ∼ 0.832)	72.00	65.00	0.37	8.52
S100B protein (pg/mL)	0.802 (0.734 ∼ 0.871)	80.00	72.00	0.52	0.44
Joint diagnosis	0.969 (0.949 ∼ 0.990	91.00	82.00	0.73	-

**Table 4:** Correlation between serum PCT, CRP, and S100B protein expression and severity of acute viral encephalitis.

Indicators	The severity of acute viral encephalitis	
	rs	*P*
PCT (ng/mL)	0.783	<0.001
CRP (mg/L)	0.769	<0.001
S100B (pg/mL)	0.745	<0.001

## Data Availability

The simulation experiment data used to support the findings of this study are available from the corresponding author upon request.
